The article "Providing an Adaptive Routing along with a Hybrid Selection Strategy to Increase Efficiency in NoC-Based Neuromorphic Systems" was published in 2021. Journal: Comput Intell Neurosci.

# Providing an Adaptive Routing along with a Hybrid Selection Strategy to Increase Efficiency in NoC-Based Neuromorphic Systems

**DOI:** 10.1155/2021/8338903

**Published:** 2021-09-15

**Authors:** Mohammad Trik, Saadat Pour Mozaffari, Amir Massoud Bidgoli

**Affiliations:** ^1^Department of Computer Engineering, North Tehran Branch, Islamic Azad University, Tehran, Iran; ^2^Computer Engineering and Information Technology Department, Amirkabir University of Technology, Tehran, Iran

## Abstract

Effective and efficient routing is one of the most important parts of routing in NoC-based neuromorphic systems. In fact, this communication structure connects different units through the packets routed by routers and switches embedded in the network on a chip. With the help of this capability, not only high scalability and high development can be created, but by decreasing the global wiring to the chip level, power consumption can be reduced. In this paper, an adaptive routing algorithm for NoC-based neuromorphic systems is proposed along with a hybrid selection strategy. Accordingly, a traffic analyzer is first used to determine the type of local or nonlocal traffic depending on the number of hops. Then, considering the type of traffic, the RCA and NoP selection strategies are used for the nonlocal and local strategies, respectively. Finally, using the experiments that performed in the simulator environment, it has been shown that this solution can well reduce the average delay time and power consumption.

## 1. Introduction

The Neuromorphic Computing, also known as “Neuromorphic engineering,” operates using a model inspired by the mechanism of the human brain. This technology not only models theories of neuroscience but also solves machine learning problems. The term neuromorphic computing is a concept developed by Carver Mead in the late 1980s describing the use of very-large-scale integration (VLSI) systems containing electronic analog circuits to mimic the neural and biological architecture present in the nervous system. Currently, the term neuromorphic is used to describe analog systems, digital systems, analog/digital complex systems, and software that model neural systems [1–3]. Interprocessor communication is supported on an effective multicast foundation managed by neurobiology. It uses a packet-switched network to achieve the very high coupling of biological systems. The packets are source-routed, i.e., they move only information near the packet issuer; the network is answerable for liberating them to their destinations. The function of a router is to be able to specify several different destinations to reach the desired packet when faced with a routing problem in sending packets. Accordingly, routers have the ability to broadcast, i.e., they can send a packet to multiple path simultaneously.

The increase in the number of components in a system on chip (SoC) coupled with the growth of interference problems caused by the bus system led to the appearance of NoC. These networks were introduced to eliminate these problems and to increase the performance of the NoC-based neuromorphic systems. In this infrastructure, instead of using wiring or communication paths, packet routing techniques are used in the network [3]. In these networks, there are several different paths to move from one node to another; therefore, there should be an algorithm to obtain the route to reach the destination. Routing algorithms may merely use the address of the current and destination nodes to compute the route (definite routing), or may use the collected traffic information of other nodes to calculate the route (adaptive routing) [4, 5]. In the adaptive algorithms, the calculated path is stored in the packet header and used in the middle nodes to hold the channels. Deadlock occurs when packets need a channel available to other packets to continue their path. Wandering also means that the packet does not arrive at the destination for long and unreasonable time. Namely, the adaptive routing algorithm measures a set of acceptable output channels regarding the paths that the packet can pass through to reach the destination [6, 7]. Afterwards, according to the network characteristics, including the congestion rate or the length of one of the routes of the output channel, the selection function will be utilized to choose the output channel from a set of permitted output channels. In this case, a traffic analyzer is used that determines the type of function according to the type of local or nonlocal traffic. As a result, in this case, according to the type of traffic, the appropriate strategy can be determined with it. The overall schematic of using the routing algorithm and selection function is presented in Figure 1 [8]. Accordingly, in this research, a hybrid function with a traffic analyzer for adaptive routing algorithms is presented, in which, in addition to increasing the efficiency of the NoC-based neuromorphic systems, power consumption can be reduced by creating the balance in this infrastructure [9, 10].

### 1.1. Contribution

In a previous work, various selection strategies have been proposed to improve routing algorithms, each of which poses challenges in research results. For example, in Ref. [11], by using a virtual circuit switch, routing is minimized and thus energy consumption is reduced. In [12–15], the selection function is presented based on the input and output choices and the NOP technique in which they have been able to reduce energy consumption.

In addition, in [16], a selection strategy is used in *XY* routing to achieve improvements in reducing latency. In the proposed method, we have first separated a number of calculations that can be done offline from the main processing steps. In this way, the processing overhead can be reduced each time it is run. In the next step, a selection strategy is presented according to the traffic situation. In this case, a traffic analyzer is used, which determines the type of selection function according to the type of local or nonlocal traffic. As a result, in this case, according to the type of traffic, the appropriate strategy can be determined with it. In this way, in addition to reducing energy consumption, other parameters such as latency and congestion can be reduced compared to other solutions.

### 1.2. Paper Organization

The study is organized as follows. In the next section, related works are stated for the previously used algorithms in NoC-based neuromorphic systems along with selection functions. In Section 3, the suggested combined method is stated to propose a combined selection function. In Section 4, the results of analyzing the suggested model in different scenarios are shown.  Section 5 concludes this paper. Finally, Section 6 discusses future works.

## 2. Related Works

Over recent years, numerous researchers have studied different utilized algorithms along with the selection functions for different fields in NoC-based neuromorphic systems, and we examine some of the performed studies in these subjects in the following sections. The neuromorphic model has scope in the development of VLSI systems, imitating the neurobiological networks of the nervous system—SNN. It is a large-scale parallel system consisting of a large number of computational units called neuromorphic nuclei interconnected by NoC. Communication management in the neuromorphic framework is the responsibility of NoC. In recent years, adaptive routing algorithms have been proposed that use local or nonlocal information for NoC. Due to the congestion of information in each router, regional congestion in NoC architectures can be divided into two categories: in some architectures, a router controls the status of the entire network, while in other architectures the routers are aware of the status of part of the network [17].

Regional congestion awareness (RCA) uses a lightweight network for accumulation and dissemination congestion information [18]. Other studies [11, 12, 19, 20] also provide information that global congestion has been reviewed and collected. Another type of architecture in neuromorphic systems that examines only a few nonlocal nodes instead of all nodes is the NoP architecture, which is based on destination-based adaptive routing. In general, the NoC architecture uses a routing strategy to avoid deadlocks. Based on the structure of NoC, two types of topology are commonly used in NoC: NoC tree and NoC mesh. Examples include NoC networks for TrueNorth and Loihi, NoC multistage networks for Dynapse [21], and NoC tree for CxQuad. SpiNNaker [13] can simulate the brain in real time by connecting 1 million ARM processors. By integrating eighteen ARM processors into a multichip processor (CMP) and 2 ^ 16 CMPs, a system with a two-dimensional network structure is formed.

In [22], a method called PACMAN is presented to study the SNN mapping in SpiNNaker. PACMAN uses a simulated annealing algorithm to search for the best partitioning plan. A variety of previous studies have examined neural network accelerators in which parameters such as reduced power consumption [23, 24], increased throughput [25, 26], and the use of memory bandwidth for information processing are evaluated. A variety of previous studies have examined neural network accelerators in which parameters such as reduced power consumption [23, 24], increased throughput [25, 26], and the use of memory bandwidth for information processing are evaluated [27]. In [9], the behavior of various topologies under the mass communication traffic of neural networks is investigated. The researchers concluded that mesh networks perform better than busses in point-to-point and tree links. Another large-scale neural network architecture is EMBRACE, which consists of a matrix of interconnected processing elements called a set of neural tiles [5]. In H-NoC, nodes are arranged in three layers, namely, module, tile, and cluster.

In the first layer, up to 10 nerve cells are connected to the router to form a neuron module. In addition, ten neuron modules are connected to the higher router to form a tile. In the higher layer, i.e., the third layer, four tiles are connected to a router, forming an EMBRACE cluster. Traffic in the neural network is multicast and all-broadcast; therefore, many previous studies that support mass communication in the NOC can be effective in managing interneuronal traffic [28]. Mass communication approaches are classified based on how the message is repeated. The main classes include single-broadcast, path-based, or tree-based multicast routing [29]. The development of processable systems is a major challenge for large amounts of multisensory data in the new age of cognitive computing. This type of intelligent computing has limitations such as real-time performance, low power consumption, and scalability. Structures and architectures imitating the brain hold great promise in this area. For this reason, in [30, 31], TrueNorth has developed a 65-megawatt real-time synaptic neural processor that uses a non-von Neumann architecture, uses low power, is highly parallel, is scalable, and is fault tolerant. NoC-enabled homogeneous CMP architectures focused on neuroscience programs that have already been explored. For example, a vastly parallelized CMP platform incorporating a custom-designed NoC architecture was used to put into effect spiking neural networks [32].

The study and analysis of neural networks in different topologies require very high configuration for these accelerators. Here are some examples of popular chips that are fast accelerators of the nervous system. Certain chips such as TrueNorth [33], Neurogrid [34], BrainScaleS [35], Loihi [32], and SpiNNaker [36] have used different features to inspire spiking neural networks. For further studies in this regard, we consider Furber solutions [16, 36] for these chips. SpiNNaker uses a processor architecture that connects to local memory on a chip. Compared to other architectures, it can be configured, but in terms of energy consumption, it is at a lower level compared to them. BrainScaleS are interconnected as several interconnected wafers, each of which consists of several HiCANN neurons. The purpose of simulating this architecture is to investigate biological neural behavior during rapid acceleration. Neurogrid is an SNN analyzer designed for analog electronics applications. This architecture operates in real time and follows several environmental methods. Finally, the architecture TrueNorth implemented in digital systems has a neuromorphic chip. These four architectures are a major step forward in the development of neural processors with the goal of mimicking the environment and reducing energy consumption in neuromorphic systems.  Table 1, by imitating Furber [16], examines the characteristics of each architecture in comparison with each other from the perspective of different parameters.

## 3. The Proposed Method

The proposed strategy that focuses on the selection algorithm develops within the framework of the infrastructure sections of these systems. Initially, the main requirements of the proposed solution are examined, and the main core of the research, which is the expression of the traffic analyzer and hybrid selection function, is presented and its capabilities are expressed. Part of the calculations of the selected strategy is done before the simulation operation; the offline execution of the calculation allows the algorithm to reduce its delay due to reduced computational time.

### 3.1. Offline Computational Strategies

Parts of the selection of computational strategies in this research, such as the link connection and the equality of resistances, are computed offline and before the algorithm is implemented, which is explained as follows:

Link contention (CL): link contention is referred to as the traffic value, which can pass through a specific link based on the communications provided in the communication graph [29]. If *p*_*i*_ is a path for arbitrary communications, *ρ*_comm_ is the set of all possible paths, *t*_comm_ is the traffic generated by communications, and *n*_comm_ is the number of all communications that are specified in the program traffic and extracted from the communication graph, the link contention CL can be expressed as follows:
  (1) $$\begin{array}{c} \text{CL}=\sum_{\text{comm}=1}^{n_{\text{comm}}}\left(µ*t_{\text{comm}}\right),\;\mu =1:\exists \rho_{i}ɛ\rho_{\text{comm}}:Lɛ\rho_{i},\text{ else}:0. \end{array}$$
Equivalent resistance (ER): by defining this concept (ER) for each given communication, and using the electrical concepts of the Kirchoff law, each node in the topology is considered as a circuit node and each link is deemed as a resistor with a volume equal to the contention of that link [37, 38].

### 3.2. Requirements of Online Function

During the execution of the algorithm, other additional available data are also used for routing, which are as follows:

(i) Free buffer rows (*d*) (*B*): the number of rows in the input buffer is the neighbors adjacent to path *d* in which *d* is one of the north, south, east, and west directions.
(ii) Instantaneous power (Δ*p*): the instantaneous power is the difference between the power consumed by the router at *t* and *t* − 1, where *t* is the moment the final output channel is selected for the packet.
  (2) $$\begin{array}{c} \Delta p=\text{power}\left(t\right)-\text{power}\left(t-1\right). \end{array}$$

Using this information, a better estimation can be obtained for the traffic load of the network and a more appropriate decision would be made at the moment of the next hop.

### 3.3. Traffic Analyzer

In order to avoid deadlock in the routing algorithm and reduce the delay time, an analyzer and selection function are added to the routing algorithm, so that it could be used to select the best outlet based on the local or nonlocal nature of the packet. Accordingly, the analyzer first extracts the destination address of each packet that is routed through the router in each *T* cycle and examines its data. For this purpose, two 5-bit counters are used to determine the local or nonlocal nature of requests in the router [14]. If the intended destination of the packet is two hops away or higher from the current router, it is considered as a nonlocal packet; otherwise, it is considered local. The analyzer calculates packet hops periodically, and accordingly, it updates the counter of locality and (*L*) and nonlocality (*N*) of the packets. This information is sent to the switcher to decide on the selection strategy. The counter is cleared at the end of every *T* cycle. The pseudocode for determining the traffic type is shown in Figure 2.

In fact, with the help of the traffic analyzer, it would be possible to obtain appropriate information about the rate of traffic and its convergence to local or nonlocal traffic [11], and then, in the next step, the routing operations can be done accordingly.  Figure 3 shows the schematic view of the solution.

Accordingly, at the end of every 32 cycles, the traffic pattern is determined by the analyzer's output, and the local traffic rate is calculated as nonlocal (*x*). If *x* ≥ 0.3, then traffic is nonuniform and the RCA algorithm [20] must be used; otherwise, the NoP [39] selection strategy will be used. In other words, if the traffic pattern is oriented towards local traffic destination, the NoP-based selection strategy is activated; otherwise, the RCA-based strategy will be activated as a proposed strategy for nonlocal traffic. The general algorithm for switching operation based on the traffic analyzer is presented in Figure 4. The data input to this algorithm is of local or nonlocal data type, and the related output is also the best strategy. It should also be noted that since the analyzer and the switch only take the router data at any one time, there is no additional overhead in network communications.

### 3.4. Formulation of the Solution

When the routing function receives multiple outputs, by reviewing the reservation table, the selected algorithm for each of these outputs checks whether the channel is available to transfer the packet (header flit) or its reserved by the other header flits [40]. The channel must be available so that the selected score is calculated, and eventually, the channel with the highest score is selected. If more channels have the same score, the first one will be chosen. The calculation of the score is done by the following formula:

(3) $$\begin{array}{c} \text{Score}\left[d\right]=\alpha \times Psel\left[d\right]+\beta \times \left(\frac{B\left[d\right]}{\max\_\text{buffer}\_\text{size}+\gamma }\right)\times \left(\frac{\Delta p}{\max\_\text{power}}\right), \end{array}$$

where *α*, *β*, and *γ* are the weight factors for the probability of selecting links, open buffers, and instantaneous power consumption. These coefficients result in the full-dynamic adaptability of the selected algorithm, and thus, the set values will be at their best state [41]. Since open buffers (*B*) and instantaneous power consumption (*p*Δ) have different units, they are normalized using max-buffer-size and max-power factors. In addition, since *Psel* is within the range (0 and 1), there is no need for normalization. Then, using the following formula, the score of the adaptive routing functions and all possible values of *α*, *β*, and *γ* are evaluated and the best coefficients are obtained for each of the routers:

(4) $$\begin{array}{c} \alpha +\beta +\gamma =1,\;\alpha =0,0.1,\ldots ,1,\beta =0,0.1,\ldots \left(1-\alpha \right),\gamma =1-\left(\alpha +\beta \right). \end{array}$$

For example, the best values of *α*, *β*, and *γ* in even-odd routing are 0.3, 0.4, and 0.3, respectively, under the MMS traffic scenario. Another important feature of this algorithm is its adaptability with any network topology [42].

## 4. Experiments and Simulation Environment

This section provides a platform for simulating the structure and framework of NoC-based neuromorphic systems. A Nirgam simulator is used to evaluate the suggested algorithm whose capabilities are listed in Table 2 [13, 19]. The main components in this simulator are routers, processing elements, links, and buffers [43, 44]. Moreover, the configuration parameters for the analysis and simulation of the suggested method are given in Table 3. In addition, the average delay, maximum delay, and power consumption are considered as the efficiency criteria. Delay is assumed as the time between entering the header flit to the network and the arrival of the tail flit to the destination node. In order to evaluate the proposed method, random, RCA, and NoP strategies have been compared [45, 46]. Here, the results of the study are shown in various traffic scenarios.

### 4.1. First Assessment: Load = 40%

In this assessment, the solutions are evaluated in the case of a traffic load of 40%. Through this assessment, the performance can be measured in low traffic and nontraffic situations. The average simulation results are achieved after 5000 runs. The evaluation results are shown in Figure 5–10. First, in Figure 5, the average overall delay in each channel is shown. As it can be observed, the proposed strategy in this case is more optimal than any other selected solutions.

Since the RCA selection strategy for a nonlocal packet has a better performance, it is, therefore, natural to lower performance in the channels; on the other hand, since the proposed strategy has different selection functions based on the length of the hop and locality and nonlocality of the channels, it has the highest efficiency. The total average delay is shown in Figure 6.

As can be seen, in total delay, the RCA efficiency increased due to the increase in nonlocal traffic rates, but given that the proposed solution core in addition to using RCA uses the NoP function for routing, naturally it has higher efficiency. In this case, the reason for this is the use of different strategies for local and nonlocal packets in which the packet will be sent with less delay and through better paths, which can lead to load balance in the network and reduce power consumption, which is clear from Figure 7.

As shown in Figure 7, the proposed solution has been able to reduce the amount of consumed power so that it is reduced by more than 50% compared to Random solution. In fact, one of the main reasons for this decrease in power consumption, in addition to offline calculations, is utilizing different strategies depending on the status of the packets, and, therefore, the best possible output path is always selected based on the network status. Accordingly, an optimal load balance is created, which reduces power consumption because in other methods such as Random, the output buffer status is not studied and, therefore, the packet may be led in a path leading to increased traffic or the placement in the queue of the input buffers of other routers, which can cause bottlenecks and increased heat and power consumption.

### 4.2. Second Assessment: Load = 70%

In this assessment, the solutions are evaluated in the case of a traffic load of 70%. Through this assessment, one can examine the performance level in a high load case. The average simulation results have been obtained after 5000 runs. The assessment results are shown in Figures 8–10.

As shown in Figure 8, although the average delay has had a significant increase in the solutions, the best output channels have been selected in the proposed solution using the selection functions that detect the local and nonlocal traffic, which results in lower delay than other solutions. The average total delay is also shown in Figure 9, and again, the optimality of the solution can be verified. Finally, in Figure 10, the power consumption is tested in the solutions and shown with a loading rate of 70%. The optimality of the proposed power consumption strategy is also well presented in this figure.

## 5. Conclusion

There are usually several different paths to move from one node to another in NoC-based neuromorphic systems; accordingly, the selection functions are used along with the routing algorithms. The effect of any routing algorithm depends on the selection strategy. When the routing function returns a set of output channels, the selection function is used to select the output channel to which the packet is sent [19]. In this research, an adaptive routing algorithm with a hybrid selection strategy is presented, and by using it and the type of traffic, it would be possible to select the best outlet channel in terms of local and nonlocal nature of the packets. Finally, in the Nirgam simulation, it was shown that this proposed method increases the efficiency significantly. The conducted tests demonstrated that this method reduces the average and maximum delay significantly compared to RCA, NoP, and Random strategies, and when some of the calculations are done offline, power consumption is reduced significantly.

## 6. Future Works

Based on the results that we have obtained in this paper, we will improve the efficiency of our method to make it more suitable for the real-world physical environment. Besides, more criteria will be taken into consideration to make our method satisfy more parallel processing in NoC-based neuromorphic systems.

## Figures and Tables

**Figure 1:** Routing structure and selection route blocks.

**Figure 2:** A pseudocode for determining the type of traffic.

**Figure 3:** The schematic view of the solution.

**Figure 4:** Pseudocode for performing switching operations.

**Figure 5:** Average total delay per channel (load = 40%).

**Figure 6:** Average total delay (load = 40%).

**Figure 7:** Power consumption (load = 40%).

**Figure 8:** Average total delay per channel (load = 70%).

**Figure 9:** Average total delay (load = 70%).

**Figure 10:** Power consumption (load = 70%).

**Table 1:** Comparison of nervous system processors in terms of structural features.

Platform	Neuromorphic system models				
	BrainScaleS	TrueNorth	Loihi	Neurogrid	SpiNNaker
NoC	Hierarchical	2D mesh	2D mesh	Tree multicast	2D mesh
Run-time plasticity	Yes	No	Yes	Yes	Yes
Implementation	Analog	Digital	Digital	Analog	Digital
On-chip learning	Yes	No	Yes	No	Yes
Neuron model	Diverse	Diverse, fixed	Adaptive quad	LIF	Fixed
Energy efficiency	Yes	Yes	Yes	No	Yes
Time	Discretized	Discretized	Discretized	Real time	Discretized
Microchip	HiCANN	EMBRACE	—	Neurocore	HiCANN

**Table 2:** Main capabilities of Nirgam simulator.

Types of production traffic	Routing algorithm type	Switching mechanism	Topology type
Constant bit rate trace and bursty based	Odd-even, *XY*	Wormhole	Torus, mesh

**Table 3:** Simulation parameters.

Parameter	Configuration
Network size	8*∗*8 mesh
Schemes	Random, RCA [19], NoP [13], proposed
Packet size	8 flits
Reset_time cycles	5000
Simulation time	10

## Data Availability

The data used to support the findings of this study are available from the corresponding author upon request.
